# Clinically Available Optical Imaging Technologies in Endoscopic Lesion Detection: Current Status and Future Perspective

**DOI:** 10.1155/2021/7594513

**Published:** 2021-02-09

**Authors:** Zhongyu He, Peng Wang, Yuelong Liang, Zuoming Fu, Xuesong Ye

**Affiliations:** ^1^Biosensor National Special Laboratory, College of Biomedical Engineering and Instrument Science, Zhejiang University, Hangzhou 310027, China; ^2^Department of General Surgery, Sir Run Run Shaw Hospital, College of Medicine, Zhejiang University, Hangzhou 310016, China; ^3^State Key Laboratory of CAD and CG, Zhejiang University, Hangzhou 310058, China

## Abstract

Endoscopic optical imaging technologies for the detection and evaluation of dysplasia and early cancer have made great strides in recent decades. With the capacity of in vivo early detection of subtle lesions, they allow modern endoscopists to provide accurate and effective optical diagnosis in real time. This review mainly analyzes the current status of clinically available endoscopic optical imaging techniques, with emphasis on the latest updates of existing techniques. We summarize current coverage of these technologies in major hospital departments such as gastroenterology, urology, gynecology, otolaryngology, pneumology, and laparoscopic surgery. In order to promote a broader understanding, we further cover the underlying principles of these technologies and analyze their performance. Moreover, we provide a brief overview of future perspectives in related technologies, such as computer-assisted diagnosis (CAD) algorithms dealing with exploring endoscopic video data. We believe all these efforts will benefit the healthcare of the community, help endoscopists improve the accuracy of diagnosis, and relieve patients' suffering.

## 1. Introduction

Endoscopy allows inspection, manipulation, and healthcare treatment of human internal organs by visualizing the region of interest minimal-invasively or even noninvasively. Since Philip Bozzini first proposed the concept of endoscopy in 1806 [1], endoscopic optical imaging modalities have got rapid developments and aid endoscopists to diagnose accurately and to reduce patients' pain.

Since the new century, the state-of-the-art optical imaging technologies in clinically available new endoscopy systems revolutionize the visualization of mucosal lesions. In order to identify early pathology and execute effective therapeutic regimens, enhanced visualization of diseased tissues is realized by utilizing the spatial-and-temporal subtle variations in tissue optical properties, such as refractive index, absorption coefficient (*μ*_*a*_) [2], scattering coefficient (*μ*_*s*_), polarization, and fluorescence properties [3]. Those subtle variations are manifested with high-contrast and high-resolution endoscopic optical imaging techniques such as narrow band imaging (NBI), autofluorescence imaging (AFI), and endocytoscopy (EC). Especially, EC even facilitates real-time in vivo optical histology.

Moreover, various research institutes have developed many other advanced endoscopic imaging systems and successfully put them into clinical use. These technologies can be classified into two categories accounting for the field of view: wide-field or microscopic-field. The first category can be further classified as wide-field white-light endoscopy (WLE) and contrast-enhancement imaging techniques. The other microscopic view category includes several existing endomicroscopy (Figure 1). Served as “red-flag” clinically available techniques, they have dramatically decreased the misdiagnosis and missed diagnosis rate and increased cure rate. In this way, they have been widely used in many hospital departments.

For this review, the PubMed and Springer Link literature search was systematically performed for studies published from 1999 to 2020 about endoscopic optical imaging technologies that have been put into human clinical use by using the search terms “Endoscopy,” “Endoscopic medical imaging and diagnosis,” “Endoscopic lesion detection,” “High-definition endoscope,” “Image-enhanced endoscopy,” “Virtual chromoendoscopy,” “Fluorescence endoscopy,” “Endoscopic special spectral imaging,” “Endomicroscopy,” “Gastrointestinal endoscopy,” “Ureteroscopy,” “Cystoscopy,” “Colposcopy,” “Hysteroscopy,” “Rhinolaryngoscopy,” “Bronchoscopy,” and “Endoscopic computer-assisted diagnosis.” Further articles were obtained through the review of the quoted references from the selected reference articles. We have included original studies that first introduced these advanced technologies and references that evaluated their clinical effect in the last few decades. Additionally, we have specially presented pieces of the literature that show current coverage of clinically available optical imaging techniques in major hospital departments, including gastroenterology, urology, pneumology, otolaryngology, and laparoscopic surgery. However, there is no once-for-all imaging modality that can be used in all clinical scenarios. Each technology has its preferred applications in various hospital departments.

## 2. A Brief Classification of Clinically Available Technologies

### 2.1. In a Wide-Field View

Endoscopists can diagnose lesions by detecting the following targets: (i) mucosal morphology (ulcer, erosion, protuberance, etc.), (ii) mucosal color (suspicious red or white spots), and (iii) vascular information (thickness, distribution, and blood concentration). In addition, according to the images of mucosal capillaries and microstructures, endoscopists can differentiate between cancer and normal because precancerous and cancerous lesions manifest significant neoangiogenesis.

#### 2.1.1. Wide-Field WLE

Recently, the imaging resolution of white-light endoscopy (WLE) reaches 1080p HD or even 4K/8K UHD (Figure 2). In addition, close focus (CF), dual focus (DF), and optical or electronic magnification bring endoscopists a clearer vision while permitting low miss rate of small lesions.

#### 2.1.2. Contrast-Enhancement Techniques

*(1) Virtual Chromoendoscopy (VCE)*. VCE augments the spatial variance of light absorption and scattering properties of tissue and organs in diagnostic and therapeutic applications. VCE has begun to replace conventional chromoendoscopy where the stain agents are necessary. VCE detects spatial variations in light absorption and scattering of the target tissue, thereby improving the contrast between abnormal and healthy tissue. According to their illumination light and image processing methods, VCE can be classified into three categories. (i) Preprocessing VCE (e.g., narrow-band imaging (NBI), red dichromatic imaging (RDI), and blue light imaging (BLI)) uses a modified spectrum light to coincide with the central peak of the absorption characteristics of hemoglobin in the blood vessels, thereby enhancing the contrast between the capillaries and the adjacent tissue from the mucosa and submucosa. (ii) Postprocessing VCE (e.g., Fujinon intelligent chromoendoscopy (FICE), i-scan, and Storz professional image enhancement system (SPIES)) processes digital image to achieve a similar effect as preprocessing VCE by spectral reconstruction algorithms. (iii) Linked color imaging (LCI) and i-scan optical enhancement (i-scan OE) which incorporate both pre- and postprocessing methods.

*(2) Fluorescence Endoscopy*. Fluorescence can provide comprehensive and detailed detection of the structure and dynamics of the targeted tissue. The fluorescence signal is wavelength dependent, and there are different fluorescent properties for different fluorophores. Thus, fluorescence spectra are often used in diagnostics [3], for it provides detailed information on fluorescence molecules, such as conformation, binding sites, and interaction within cells and tissues [4]. In addition, the fluorophores can be further divided into endogenous fluorophores or exogenous fluorophores. With customized optical filters blocking the false excitation light to a sufficiently low level, sensors in fluorescence imaging optical systems capture part of the emitted fluorescence from the tissue and contribute to the final images [3]. The existing clinically available fluorescent endoscopy system includes autofluorescence imaging (AFI), near-infrared imaging with indocyanine green (IRI and NIR/ICG), and photodynamic diagnosis (PDD). AFI uses violet light to excite endogenous fluorophore, while NIR/ICG and PDD use a modified range of light to excite exogenous fluorochrome applied to the region of interest.

Nevertheless, these contrast-enhancement techniques stated above have different working wavelengths and penetration depths (as shown in Figure 3 and Table 1). They all have been well applied in various departments according to their technical characteristics.

### 2.2. In a Microscopic View

With the aid of the endocytoscopy (EC) or confocal laser endomicroscopy (CLE) which enables real-time micron-level imaging, endoscopists can characterize the suspicious lesions by visualizing the following microstructural objects: multicellular structure such as capillaries, villiform structure, cellular morphology as crypt, goblet, or epithelial cells, and subcellular organelles (nucleus and cytoplasm). Thus, EC and CLE systems are able to allow in vivo “optical biopsy” and are promising to supersede place ex vivo histology which is the current gold standard for endoscopic diagnosis. Furthermore, they can be integrated into the distal end of the conventional WLE, facilitating endoscopists to visualize the mucosa from both wide-field and microscopic views in the meantime.

Table 2 points out the advancements and existing shortcomings of each technology. Some latest technologies demand more clinical experimental data to evaluate their clinical performance more thoroughly. Furthermore, Figure 4 shows the timeline of their clinical use and their corresponding clinically available endoscopic systems. All of the advanced endoscopic imaging technologies have been put into clinical use in the last 20 years.

## 3. Optical Imaging Technologies in Major Hospital Departments

In this section, we introduce clinically available technologies by hospital departments.  Table 3 generally summarizes the coverage of each technology in different departments.

### 3.1. In Gastroenterology

Advanced endoscopic imaging technologies such as VCE and fluorescent endoscopy play an essential role in the detection of gastrointestinal (GI) diseases, especially superficial mucosal lesions. In the esophagus, they enhance the visualization contrast between capillary and surrounding tissue. Thus, the morphology of intra-epithelial papillary capillary loop (IPCL) can be analyzed for evaluating the tumor invasion according to the Japanese Classification of Esophageal Cancer by the Japan Esophageal Society (11th edition) [5]. As for the stomach and colon, lesions are diagnosed by visualizing the microvascular patterns (microvascular patterns can be classified into the following five groups: mesh, grid, spiral, loop, and branch) [6] and microstructures on the mucosal surface (e.g., glandular ducts, capillaries, and villus). VCE can also help propose correct and valid treatment methods. Moreover, EC and CLE are able to diagnose various GI diseases by detecting the crypt structures, villiform structures, the morphology of small vessels, goblet cells, epithelium cells and their organelles (nucleus), etc.  Figure 5 shows the development history of endoscopic diagnostic tools in gastroenterology.

#### 3.1.1. Wide-Field HD-WLE

Radiating a broad spectrum of visible white light from a xenon lamp or light-emitting diodes (LEDs), white-light endoscopy (WLE) can image the mucosa with true to life representation. High-definition (HD) video endoscopes already use charge-coupled devices (CCDs) or complementary metal oxide semiconductor (CMOS) to produce images with a resolution of more than one million pixels. Monitors display HD images usually with 4 : 3 or 5 : 4 aspect ratios and at least 650–720 pixels in height [7]. In addition, surface details including pit patterns and vascular structures can be further enhanced when combined with zoom lenses, which can magnify images by up to 150 times [8].

Ultra-high definition (4K UHD) offers 3840 × 2160 pixels and wide color gamut in Bt. 2020. However, UHD has not been realized in chip-on-tip gastrointestinal endoscopes until now, due to the challenge of designing the high-quality objective lens and high-speed data transmission.

#### 3.1.2. CF and DF

Close Focus (Olympus and Fujifilm, Japan) are achieved by optimizing the structure of the lens integrated into the distal end of the endoscope. The fixed close focusing system decreases the minimum visible length to 2 mm from 3 mm from the distal end (Figure 6). Endoscopes with close focus examination range allow endoscopists to get closer to the mucosa for even higher resolving power and magnified visualization of the tissue and capillary networks. In this way, endoscopists can obtain more information on the mucosal surface which can not be obtained by electronic magnification.

Dual focus two-stage optical lens technology allows endoscopists to switch from normal focus mode to near focus mode with a single button so that they can conduct a close examination of mucosal tissue and capillary networks. The field depth of normal and near focus mode, for example, is 7–100 mm and 3–7 mm, respectively. This new technology lets endoscopists select the desired depth of field and obtain high-quality images at the same time, which brings a new level of visualization to routine examinations [9]. Thus, diagnostic accuracy can be improved [10–13].

#### 3.1.3. NBI

Narrow band imaging (NBI) may become the most widely used optical imaging technique [14]. Compared with traditional stain-based chromoendoscopy, NBI provides higher contrast without the use of dyes. Two electronically activated filters were placed in the light path to limit the full spectrum of visible white light to a center wavelength of 415 (blue) nm and 540 nm (green) [15] (as shown in Figure 7). These wavelengths coincide with the central absorption peak of hemoglobin (maximal at 415, 542, and 577 nm for oxyhemoglobin, and 430 and 555 nm for deoxyhemoglobin [16]), so certain histological structures with high hemoglobin content such as capillaries and veins are represented darker, which provides a contrast to the surrounding mucosa that reflects light. Capillaries in the superficial mucosal layer are accentuated by the 415 nm light and are displayed in brown, whereas submucosal vessels buried in deeper mucosal are made visible in cyan by the 540 nm light. The composite NBI images are displayed by feeding the 415 nm image in the blue and green channels and the 540 nm image in the red channel of the monitor [17]. The NBI mode can be activated by simply pressing a button on video endoscopy systems, allowing for rapid alternation between NBI and WLE [15, 18].

Therefore, NBI owns the ability to reveal essential features clearly. It not only emphasizes surface microvasculature but also enhances the boundary between different types of tissue [19]. NBI represents a major step forward for the detection and characterization of GI lesions, especially neoplasia. Also, it has been used in grading esophagitis [20], the identification of Barrett's esophagus [21], the identification of pit patterns to classify colorectal polyps and tumors [22], and the detection of atypical dysplastic tissue in the colon of patients with ulcerative colitis [23].

Furthermore, NBI can reduce the times of biopsies due to more mucosal information can be provided. However, there seems to be little evidence to justify the routine use of the initial NBI system because of its low illumination intensity. The lack of lighting leads to dimmer imaging, especially in the case of the stomach and colon cavity. In 2013, to overcome the above issue, the second-generation NBI endoscopy systems (*EVIS LUCERA ELITE* and *EVIS EXERA III*, Olympus) have been providing a higher illumination intensity by optimizing the light source, optical filters, and fiber transmittance to achieve the best possible images for early dysplasia detection and improve procedural efficiency [24]. Most recently, in the latest endoscopic system (*EVIS X1*), Olympus directly adopted two LED lights with specific central wavelengths of 460 nm and 540 nm, respectively, to provide narrow band light (third-generation NBI, as shown in Figure 8), which could extend the life of the light source and reduce the volume of the system in contrast to the previous series.

However, some researchers argue that compared with HD-WLE, NBI does not increase the detection of colon polyps, adenomas, or flat adenomas. Also, it does not decrease the miss rate of colon polyps or adenomas in patients undergoing screening/surveillance colonoscopy [25]. In addition, NBI was reported to have no additional benefits over WLE at screening colonoscopy for nonexperts [26]. Hence, multicenter clinical trials with consistent criteria are needed to verify the effectiveness of the NBI and to optimize the interoperator performance.

#### 3.1.4. RDI

Red Dichromatic Imaging (RDI), also called dual red imaging (DRI), is a novel image-enhanced endoscopy technique, which was designed to enhance the visibility of blood vessels and bleeding sources in deeper tissue by using narrow-band light at two center wavelengths in the red band: 600 and 630 nm [27, 28]. These wavelengths are able to detect thick blood vessels at a depth range of 1,000–1,500 *μ*m from the mucosal surface of the gastrointestinal wall [29], and they are between the wavelength of 576 nm (at which the light absorption coefficient reaches the maximum of the light absorption property of hemoglobin) and the wavelength of 730 nm (at which the light absorption coefficient reaches the minimum of the light absorption property of hemoglobin). Moreover, the light absorption of blood vessels at 600 nm is much stronger than that at 630 nm [29]. RDI utilizes green, amber, and red wavelengths to visualize bleeding points or deep blood vessels [28] (Figure 8). Once the amber light (600 nm) hits the above targets where the blood concentration is very high, the amber light is strongly absorbed. Thus, bleeding points or deep blood vessels appear darker and are therefore more visible because the color difference between them and surrounding tissue was clear [30].

In this way, RDI helps to efficiently identify the bleeding source during endoscopic resection treatments which make hemostasis quicker and easier. In addition, DRI has the potential to gain clear endoscopic visibility during colorectal ESD, especially with submucosal fatty tissue [31, 32]. Therefore, RDI helps to reduce stress and procedure time for the treatment of emergency bleedings and endoscopic resections [33]. Kubosawa et al. [27] firstly reported the usefulness of DRI for attaining hemostasis in a case with bleeding from a gastric ulcer in which the bleeding point was difficult to identify by WLI, which indicated DRI has the potential to simplify hemostatic treatment for gastric ulcer bleeding [30]. Furuichi et al. [28] found that DRI increased the visibility of the esophageal varices (EVs) and red color sign (RCS); especially, EVs or RCS in the shallower position was more enhanced by DRI. And, visual recognition of the changing degrees of visibility by DRI enables the prediction of the depth of esophageal varices.

Moreover, RDI can visualize the inflammation, including that in the surface crypt, and vessel findings of the brownish surface or green-colored deeper layer of the mucosa in contrast to NBI. Moreover, as a practical approach, RDI has potential in the evaluation of histological inflammation and assessing the severity of inflammation without the requirement of a biopsy in patients with ulcerative colitis [34]. The prognosis of ulcerative colitis can be predicted by assessing deep vessels using DRI [35].

#### 3.1.5. BLI

Blue light imaging (BLI) focuses on the light absorption characteristic of hemoglobin (at 410 nm). By combining violet light with the specific white light, BLI can improve color contrast of mucosal images. Instead of xenon light whose life expectancy is quite short (500 hours in usual), the light spectrum of *ELUXEO* systems is emitted by the optimal combination of 4 LEDs (∼60,000 hours). The light spectrum of the system has specific peaks at 400 nm (violet light) and 450 nm (blue light), which highlights the contrast between blood vessels and surrounding tissues by using the same principles as NBI (Figure 9). In addition, by concentrating and intensifying specific wavelengths of illumination, BLI can get a better visualization of the superficial microvessels and mucosal surface structures to enhance the subtle contrast of the irregularities of the mucosa with a safe diagnostic and therapeutic procedure [36], especially in diagnosing the colorectal polyps in GI tract [37–39].

#### 3.1.6. FICE

Fujinon intelligent chromoendoscopy (FICE) is similar to i-scan [40]. As another *post*processing virtual chromoendoscopy, FICE uses image enhancement algorithms based on spectral estimation from RGB values [41] recorded by the CCD. In this way, white-light images are digitally converted into color images composed of three specific virtual single-wavelength images that are randomly selected and assigned to the red, green, and blue. By combining the three channels, the color image can enhance the visualization of mucosal structures and microcirculation. In addition, endoscopists can select 60 spectral images per 5 nm at visible wavelengths (400–695 nm) and set up five gradations of spectral image intensities. There are ten available presets that can be customized and configured from the many possible permutations [15], and an appropriate setting is chosen based on the targeted lesion characteristics [42]. Like the NBI system, FICE images can be magnified optically and digitally. However, there is a tendency that FICE is not utilized in newly released endoscopy systems developed by Fujifilm because BLI and LCI own better visualization of the target lesion and clinical diagnosis accuracy [43].

#### 3.1.7. SPIES

Recording video within an RGB camera of the modular IMAGE1 S platform, the Storz professional image enhancement system (SPIES) is a novel technique capable of enhancing the appearance of the mucosal surface. SPIES adapts color processing algorithms to amplify the spectral separation [44]. It owns several different visual-digital reprocessing imaging modes such as Clara, Chroma, Clara + Chroma, Spectra A, and Spectra B [45], which can be used to modify the displayed mucosal video images and increase viewing comfort for the endoscopists. Among these modes, Clara provides homogeneous illumination with clear visibility of darker regions due to the adaptation of local brightness, while Chroma increases the contrast of the images to enhance the structures within the displayed image. The rest of the modes are SPECTRA A and SPECTRA B, which shift and exchange the image effective spectral response, highlighting the contrast between different tissues and structures [44] related to different penetration depths [46] (Figure 10). All these five modes are potential candidates to choose the best option according to the specific clinical situation. For instance, the Spectra B is suggested in case of interference such as in hematuria, whereas the Spectra A is suggested in case the surgeon desires a higher contrast of the image [47]. However, the SPIES is relatively new (Figure 4), and the clinical value of the system is currently under investigation [48].

#### 3.1.8. I-Scan OE

I-Scan Optical Enhancement (I-scan OE) is an updated technology based on i-scan (Figure 11) which is a digital contrast method comprising three modes (surface enhancement (SE), contrast enhancement (CE), and tone enhancement (TE)) that involves postprocessing software applied on white-light images [49, 50]. I-scan OE creates a more progressive platform where both digital and optical enhancements are available. The combination of bandwidth-limiting light with digital image processing provides extra information for a more accurate in vivo diagnosis through the improved vessel and mucosal pattern characterization.

In order to obtain microvascular pattern images with higher contrast, i-scan OE changes the conventional white-light illumination by placing optical filters in front of the light source. The newly designed optical filters are able to achieve higher overall transmittance by connecting the peaks of the hemoglobin absorption spectrum (415 nm, 540 nm, and 570 nm), which creates a continuous wavelength spectrum and raising baseline transmittance between these absorption peaks. By maximizing the amount of illumination, the darkness when detecting the GI lumen in wide-range observation can be overcome [51]. Thus, I-scan OE is promising to decrease the miss rates of lesion detection and increase the accuracy of characterization, which offers new potential for enhanced diagnosis of lesions throughout the whole luminal GI tract. [52].

#### 3.1.9. LCI

Based on blue light imaging (BLI), linked color imaging (LCI) is capable of emphasizing slight color differences and provides a better color contrast within the red color range by utilizing an advanced image processing algorithm with optimal illumination light. Consequently, the originally red regions become a deeper shade of red, and originally white areas appear brighter while natural tones still exist [53]. As a result, the increased color contrast leads to a more accurate delineation and earlier detection of lesions and inflammation than the conventional WLE [54–56].

#### 3.1.10. AFI

With the aim to detect neoplastic lesions, autofluorescence imaging (AFI) is based on the excitation of endogenous fluorophores in the tissue, such as collagen, elastin, and flavins. Excited by a specific shorter wavelength, these endogenous fluorophores emit autofluorescence with longer wavelength accordingly. After the occurrence of adenomas or neoplasms, the increase in the thickness of the mucosal layer reduces the autofluorescence output from the submucosa. Therefore, the tissue morphology and structure will alter the endogenous fluorescence spectrum. Consequently, healthy and abnormal tissue regions have diverse emission spectra under AFI [57].

A rotating filter placed in front of the xenon arc lamp generates the blue excitation light (390–470 nm) and green light (540–560 nm). These fractionated lights are radiated sequentially during AFI endoscopy. Another interference filter placed in front of the monochrome CCD removes reflected excitation light. However, both autofluorescence and green reflectance light from the mucosa with the range of 500–630 nm can travel through the filter selectively. The AFI system produces a single pseudocolor image by allocating the autofluorescence signal to the green channel while the reflected green light to the red and blue channels at 1 to 0.5 ratio to show normal mucosa as green and dysplastic/cancerous tissue as magenta or purple in color (as shown in Figure 12).

The currently available AFI system (*EVIS LUCERA SPECTRUM*) with trimodal (WLE + NBI + AFI) capability has two separate CCDs for WLI and AFI. One CCD is for high-definition WLE and NBI, and the other CCD is specific for AFI [58]. Because the autofluorescence is relatively weak, newly developed high-sensitivity CCD can accurately detect the fluorescence, making it possible to discover subtle differences in mucosal structures and adenomatous lesions that would be difficult to detect in WLE [59].

However, the image resolution of AFI is even lower than WLE, for frame averaging is utilized to increase the quality of the autofluorescence image, and the intensity-based contrast of AFI is often not sufficiently specific [60, 61]. In addition, the quick movement of the endoscope distal tip leads to the degradation of the images as the frame averaging cannot keep pace [62].

#### 3.1.11. IRI

Unlike VCE, which can only obtain diagnostic information from the surface of mucosa and the middle layer of mucosa, infrared imaging is able to detect the deeper layer of mucosa by irradiating two bands of near-infrared light (790–820 nm and 905–970 nm) following intravenous injection of indocyanine green (ICG). ICG strongly absorbs the NIR light and emits the fluorescent light. Therefore, the contrast-enhanced images of the vessels deep in the mucosa can be clearly displayed. Also, the IRI system can monitor blood flow. Thus, IRI could be helpful to determine a therapeutic strategy which relies on the degree of invasiveness of cancer.

Officially launched in 2007, the *LUCERA SPECTRUM* is the first endoscopic system that integrates IRI (Figure 4). The system also includes other several modes: NBI, AFI, and WLE. In 2013, the new-generation system called *EVIS LUCERA ELITE* still reserved IRI mode (Figure 13).

IRI has already been investigated in examinations of the upper GI tract for medical efficacy. For instance, Mataki et al. [63] first showed that IRI provides valuable information about the degree of invasiveness of early gastric cancer. In addition, Nakayoshi et al. [64] proposed that the IRI System may predict delayed-type bleeding from the mucosal defect after EMR (endoscopic mucosectomy) or ESD (endoscopic submucosal dissection) for the gastric tumors. In this way, IRI may become a useful technique for determining whether to perform EMR or ESD shortly [65]. In addition, IRI can be used to detect the depth of cancer and assessment for therapeutic measures.

#### 3.1.12. EC

Endocyto (EC) is a kind of ultra-zoom endoscopy which has presented a new era of diagnosis. It equips with a manual zoom mechanism resembling a conventional magnifying scope. Based on the principle of contact white-light microscopy with a fixed-focus, high-power objective lens project ultra-high image from target region on to a charge-coupled device at a frame rate of 30 Hz [66]. Thus, EC enables real-time in vivo visualization of the cytological structures of the superficial epithelial layer in a plane parallel to the mucosal surface in cellular and even subcellular level. After removing the excess surface mucus [67], an appropriate dye (e.g., methylene blue, toluidine blue, and cresyl violet) [68] stains the cell nuclei. Then, the light emitted by the light guide is sent into the cells and partially returned as scattered light, facilitating observation of the architectural features, such as the size and shape of cells, nuclei, and the nucleus to cytoplasm ratio [68, 69]. Depending on these features, EC allows endoscopists to accurately distinguish single inflammatory cells, namely, basophilic or eosinophilic granulocytes and lymphocytes. Furthermore, concordance between endocytoscopy and standard histopathologic grading of disease activity is 100%, and EC exhibits a substantial interobserver and almost perfect intraobserver agreement [70].

There are two types of available endocyto. One is endoscope-integrated endocytoscopy (eEC, 580-fold magnification) while the other is probe-based handheld endocytoscopy (pEC, 570-fold magnification, or even up to 1390-fold magnification) [70]. In addition, a new endocytoscopy system with continuous zooming to a 400-fold magnification is also reported [71]. The axial resolution of endocyto systems varies from 0–50 *μ*m, while the lateral resolution of ultra-zoom endoscopes varies from 1.7–4.2 *μ*m [68]. Also, endocyto incorporates a broad range of observation modalities, including magnifying NBI under the system of *EVIS LUCERA ELITE* to access the lesion in the GI tract. Thus, the color contrast under the magnified view is enhanced.

Recent studies have shown that endocytoscopy has the potential to change the current paradigm for the diagnosis of GI diseases [71]. However, vital staining is relatively poor in the stomach because of gastric secretions and inflammatory products which make endocytoscopic observation more difficult than elsewhere in the GI tract. Hence, studies on endocytoscopic observation of the stomach have been limited [72].

#### 3.1.13. CLE

Confocal laser endomicroscopy (CLE), similar to bench-top confocal laser scanning microscopy, works by focusing laser light through a single lens onto a specific focal plane of the target tissue. CLE is a groundbreaking tool for translational science for understanding epithelial regulation and pathophysiology. Spatial filtering is the fundamental basis of confocal imaging. The term confocal refers to the alignment of both the illumination and collection systems in the same focal plane [73, 74]. The laser light is focused through a pinhole at the selected depth, and reflected light is then refocused onto the detection system by the same lens. Thus, the point of illumination coincides with the point of detection within the specimen. In this way, the light reflected and scattered at other geometric angles from the illuminated object as well as out-of-focus light are rejected by the pinhole and do not reach the detector (Figure 14).

Generally, in order to obtain a strong fluorescence signal, the size of the pinhole should be set to be equal to the size of the Airy spot of the system. Moreover, by reducing the size of the pinhole, the theoretically ultimate lateral (*x*, *y*) and axial (*z*) spatial resolution of confocal imaging are

(1) $$\begin{array}{c} d_{x,y}\approx \frac{0.4\lambda }{\text{NA}}, \end{array}$$

(2) $$\begin{array}{c} d_{z}\approx \frac{1.4\lambda n}{{\text{NA}}^{2}}, \end{array}$$

where NA is the numerical aperture of the objective, *λ* is the wavelength of incident laser light, and *n* is the refractive index of the medium between objective and tissue.

Furthermore, the main advantage of CLE is its optical sectioning ability (that is, multiple “slices” through the tissue, a so-called *z* stack) [75]. The CLE can give insight into the three-dimensional tissue structure and provide a real-time in vivo histological diagnosis with gray-scale images presented a high spatial resolution [76] (as shown in Figure 15). By integrating a miniature scanner onto the endoscope tip, confocal scanning was performed at laser illumination for excitation of exogenously applied fluorophores (topical acriflavine [76] and intravenous fluorescein [77]) in order to contrast cellular, subcellular, connective tissue, and vessel architectures in clinical studies. Furthermore, CLE is theoretically possible to use autofluorescence for imaging [73, 74, 78].

There are two kinds of FDA-approved and CE-certified devices which are available to perform CLE: endoscope-based CLE (eCLE) and probe-based CLE (pCLE).  Table 4 summarizes the property of eCLE and pCLE [79]. The eCLE system is integrated into the tip of the conventional endoscopes, while pCLE involves kinds of microprobes that can be inserted into the accessory channel of gastrointestinal endoscopes for minimally invasive imaging (as shown in Figure 16). In comparison, the main advantage of eCLE over pCLE is that the imaging plane depth of eCLE is adjustable because its laser scanner is integrated into the distal tip of the endoscope. In addition, eCLE allows the optical sectioning of the tissue with a higher axial resolution. Its maximum scanning depth is up to 250 mm. Nevertheless, the frame rate of pCLE is much higher than that of eCLE. And, pCLE can bridge the gap between wide-field detection and microscopic characterization when it combines with wide-field WLE to unmask suspicious areas. Both eCLE and pCLE are capable of visualizing the mucosal layer of the GI tract with a subcellular resolution during ongoing endoscopy [80].

Recently, Mauna KeaTech developed a pCLE system that presented tissue images in two colors (red and green) by introducing two excitation wavelengths (488 + 660 nm). In this way, the system can further improve image contrast and provide more diagnostic information.

However, CLE still has limitations: (i) the low imaging frame rate and the presence of moving artifacts prevent proper and quick 3D reconstructions during endomicroscopy [81]; (ii) applying fluorescence agents increases the whole procedural time; (iii) the toxicity of fluorescence agents is also need to be taken into further consideration, for instance, the acriflavine is a carcinogenic dye [82], so its clinical utility should be evaluated prudently [78]; (iv) the difficulty in interpreting the acquired image leads to the interobserver and intraobserver variability [83]; (v) the relatively higher purchase and maintenance costs and limited lifespan will influence the cost-effectiveness of the CLE system [78].

#### 3.1.14. The PIVI threshold

For a long time, no evaluation standard or a technical threshold existed to judge whether any endoscopic imaging techniques could be clinically used in the detection of various GI diseases. However, in 2015, the American Society for Gastrointestinal Endoscopy (ASGE) Technology Committee proposed the Preservation and Incorporation of Valuable endoscopic Innovations' (PIVI) thresholds for adopting real-time endoscopic assessment of the histology of diminutive colorectal polyps [84]. There are two thresholds have been established in this PIVI paper:

1. For a technology to be used to guide the decision to leave suspected rectosigmoid hyperplastic polyps 5 mm or smaller in place (without resection), the technology should provide a 90% or higher negative predictive value (when used with high confidence) for adenomatous histology
2. For colorectal polyps 5 mm or smaller to be resected and discarded without pathologic assessment, endoscopic technology (when used with high confidence) used to determine histology of these polyps, when combined with the histopathologic assessment of polyps larger than 5 mm, should provide 90% or higher agreement in assignment of postpolypectomy surveillance intervals when compared with decisions based on pathology assessment of all identified polyps [84]

However, although magnifying chromoendoscopy, narrow-band imaging (NBI), endocytoscopy (EC), and confocal laser endomicroscopy (CLE) are highly accurate for the detection of diseases, interpretation of these modalities is difficult for novices. Hence, achieving a negative predictive value of >90% for adenoma is relatively difficult to use these modalities and requires comprehensive experiments [85].

Similarly, the ASGE Technology Committee also proposed thresholds for adopting real-time imaging-assisted endoscopic targeted biopsy during endoscopic surveillance of Barrett's esophagus [86]. The committee suggests that such a technique should have a 90% per-patient sensitivity, 80% specificity, and 98% or greater negative predictive value (NPV) for detecting high-grade dysplasia (HGD). However, as far as we know, there have been no criteria or thresholds to judge any optical imaging technology's acceptability in the diagnosis of other diseases except the above two thresholds. Thus, more thresholds need to be put forward to evaluate the application value of kinds of endoscopic imaging techniques in gastroenterology.

### 3.2. In Urology

White-light endoscopy has been used in urology for more than 100 years. For a long time, the combination of white-light cystoscopy and ex vivo biopsy has been the “gold standard” for the diagnosis of urological cancer. However, the traditional method cannot effectively identify small papillary cancer, early squamous carcinoma in situ (CIS), atypical hyperplasia, flat urothelial lesions, and so on, thus increasing the residual or recurrence of tumors after surgery. The emergence of advanced endoscopic imaging technologies below can help improve the accuracy of the diagnosis of urinary tract diseases.

#### 3.2.1. NBI

In recent years, the application of NBI endoscopy has made rapid progress in the diagnosis, treatment, postoperative monitoring, and follow-up of urothelial diseases. NBI can improve the detection rate of urothelial tumors, provide more accurate tumor margins, and facilitate the early detection and diagnosis of microscopic lesions [87]. Compared with a white-light cystoscopy, NBI cystoscopy is more sensitive to diagnose interstitial cystitis (IC). The positive area detected by NBI cystoscope is highly consistent with the positive area detected by water dilatation test, which is of high application value for the diagnosis of IC [88]. Byran et al. [87] reported that NBI technique could detect lesions that could not be detected by conventional white-light cystoscopy. In addition, NBI cystoscopy improves the detection rate of primary and recurrent nonmuscle invasive bladder cancer (NMIBC) over white-light imaging (WLI) [89].

Moreover, compared with traditional white-light ureteroscopy, NBI ureteroscopy could accurately display the boundary between tumor tissue and normal renal pelvis or ureteral mucosa, which significantly improved the detection rate of urothelial tumors in the upper urinary tract [90]. In addition, Olivier et al. [91] performed NBI and white-light flexible ureteroscopy in 27 patients and found that NBI could provide more detailed boundaries and vascular architectures of upper urinary tract transitional cell carcinoma. In their experiment, NBI improves the tumor detection rate by 23% compared with WLE.

#### 3.2.2. SPIES

The Storz professional image enhancement system facilitates the treatment of bladder cancer by providing more explicit mucosal images. It was reported that SPIES is able to reduce the number of tumors missed by gold standard WLI [92]. Moreover, once endoscopists find a tumor, SPIES can help them find the demarcation between the tumor and healthy tissue, thus removing the tumor more completely. By obtaining a complete excision, the use of SPIES is expected to reduce the recurrence rate, which means patients need a less invasive diagnosis and surgical treatment [93]. Kamphuis et al. [94] evaluated the variation of interpretation of the same bladder urothelium image in different SPIES modalities. They found that images in Spectra B had less variation in interpretation than WLI and Spectra A. The image quality in SPIES modalities was graded significantly higher than WLI.

#### 3.2.3. PDD

Photodynamic diagnosis (PDD) involves fluorescence to localize lesions. Therefore, PDD is also known as fluorescence diagnosis or fluorescence photodetection. The diagnostic value of PDD depends on the selective accumulation of fluorochrome and on how well interfering optical tissue inhomogeneities can be considered or eliminated [95]. By implying a contrast in fluorescence of diseased tissue versus healthy tissue, PDD can reveal neoplastic lesions that cannot be seen by WLE.

In urology, PDD is mainly focused on improving the detection rate of hardly visible urothelial bladder cancer. The principle of cancer recognition is based on the abnormal metabolism of tumor cells in the process of heme synthesis. PDD requires preoperative intravesical instillation of fluorophores that are taken up by the urothelium and preferentially metabolized by abnormal cells. Unlike AFI, PDD generally uses exogenous fluorophores. After injection of 5-aminolevulinic acid (5-ALA) or hexaminolevulinate (Hexvix), a fluorescent substance, protoporphyrin IX (PpIX), is produced and accumulated in the tumor cells. PpIX is red by PDD technology. Thus, the tumors (red) and surrounding tissues (blue) can be clearly identified.

Among several exogenous fluorochromes, the Hexvix has obtained approval for the detection of bladder cancer in 26 European countries. They are activated by the light in the appropriate range, and then, they emit fluorescence. According to the 2006 European Association of Urology (EAU) guidelines, PDD has been accepted as a method to reveal areas in the bladder that are suspicious of carcinomas in situ (CIS) or of developing a papillary tumor [95]. German corporations such as Richard Wolf and Karl Storz have already launched mature cystoscopy products with PDD.

Furthermore, reports also showed promising results of PDD for the detection of urethral human papillomavirus (HPV) lesions [96], prostate cancer [97], and kidney tumors [98].

#### 3.2.4. EC

Ohigashi et al. [99] used a probe-based EC system with 450-fold magnification to evaluate bladder carcinoma in five patients. The probe was inserted into the working channel of a rigid cystoscope. As a result, the cell structure and nuclear morphology of the bladder tumors were identified and graded with an accuracy of 80%.

#### 3.2.5. CLE

Confocal laser endomicroscopy can also be used to detect urological lesions. In contrast to standard pathologic analysis of fixed tissue with hematoxylin and eosin, pCLE (*UroFlex* and *CystoFlex*, Cellvizio, Mauna Kea Tech) provides real-time visualization of the urinary tract under a microscopic view to enable dynamic interrogation of benign and neoplastic tissues in vivo. Wu et al. [100] proposed the confocal diagnostic imaging criteria for normal, inflammatory, low, and high-grade cancer, which might facilitate the adaptation of pCLE in conjunction with white-light cystoscopy to expedite diagnosis of urinary tract pathology, particularly the bladder cancer. Furthermore, CLE can characterize optical imaging features of healthy, benign, and malignant prostate [101].

### 3.3. In Gynecology

Pathologically, endometrial hyperplasia is classified as simple hyperplasia, complex hyperplasia, and atypical hyperplasia, which is recognized as a precancerous lesion of endometrial cancer. Studies have shown that the occurrence and development of tumors depend on angiogenesis, and the intensity of angiogenesis has a predictive effect on the diagnosis of malignant tumors. Moreover, research showed that the sensitivity of conventional WLE to endometrial hyperplasia and endometrial cancer was only 56.3% and 80% [102]. Therefore, it is not sufficient to diagnose endometrial lesions merely by observing the morphological changes of the uterine mucosa. The application of the following technologies will improve the above situation.

#### 3.3.1. NBI

With an outstanding ability to detect capillaries, NBI hysteroscopy can improve the diagnostic sensitivity of endometrial cancer and endometrial hyperplasia with high diagnostic specificity and high consistency to histological results [103]. It was also reported that NBI had promising progress in diagnosing cervical adenopathy [104].

#### 3.3.2. SPIES

The SPIES is a helpful modality to target strip biopsies. According to the clinical experiment carried out by Schneider et al. [105] in 102 patients, the trauma/pain perception can be decreased while maintaining diagnostic accuracy in patients with the diagnosis of high-grade squamous intraepithelial lesions of the uterine cervix.

#### 3.3.3. PDD

3% 5-ALA was used as a photosensitizer to detect cervical intraepithelial neoplasia with higher sensitivity than white-light colposcopy and higher specificity than the cytological diagnosis. Furthermore, PDD allows for the precise location of a cervical neoplastic change as well as its extension, borders, or multifocal character [106].

### 3.4. In Otolaryngology

Most malignant tumors in the head and neck are associated with the local invasion into adjacent organs, which will significantly increase the mortality rate of cancer patients and affect their quality of life. Therefore, early detection, diagnosis, and intervention of cancer are problems to be solved in clinical work. The endoscope is a useful instrument for the diagnosis and treatment of malignancies originating from the head and neck region. However, WLI has technical limitations in detecting small or superficial lesions on the mucosa [107]. However, the innovative and noninvasive electronic endoscopy imaging technologies below can break this limitation.

#### 3.4.1. UHD-WLE

Rigid sinuscopes with Full 4K resolution have been put into clinical use in the last few years [108, 109]. By providing UHD video imaging systems, the operation visibility is equivalent to open surgery for the detection of ear, nose, and throat lesions. Imaging with Full 4K can display four times more detail than Full HD, and immersive experience with a closer distance can be provided. In addition, a wider color gamut is provided to realize rich color reproduction for the video recorded by the system. Recently, 4K technology helped endoscopists investigate oral and oropharyngeal squamous cell carcinoma [110], Cholesteatoma and Otosclerosis surgery [111], etc.

#### 3.4.2. NBI

Compared with the widespread use in the digestive system, NBI is just beginning in the field of otolaryngology, head and neck surgery, and has made some progress which mainly focusing on the examination of throat tumors. The sensitivity and specificity of NBI in the diagnosis of malignant laryngeal lesions were higher than that of conventional white-light electronic rhinolaryngoscopy [112]. Xiaoguang et al. [113] analyzed the morphological characteristics of microvessels on the mucosal surface of 240 patients with nasopharyngeal lesions of different properties. They found that the neovascularization on the surface of nasopharyngeal carcinoma lesions under NBI mode was tan and clear, with the appearance of thin dendritic or twisted lines. Thus, NBI showed the special significance in the diagnosis of nasopharyngeal carcinoma, and its sensitivity to the disease reached 80.6%, while the specificity, positive predictive value, and negative predictive value were 91.7%, 96.7%, and 61%, respectively. Thus, it is believed that NBI can improve the role of endoscopy in the early diagnosis of nasopharyngeal carcinoma. The recommended IPCL classification system (2011) has played a positive role in promoting the research of NBI in this field [114]. The IPCL predicted that NBI will have a broad prospect in the application of nasopharyngeal cancer, hypopharyngeal cancer, laryngeal cancer, and other malignant tumors. However, the clinical value of NBI in head and neck tumors still needs more scientific and objective studies.

#### 3.4.3. SPIES

More recently, the Storz Professional Image Enhancement System was reported to succeed in identifying significant epithelial and subepithelial microvascular changes in larynx and hypopharynx, especially in the Clara + Chroma and Spectra A/B modes [45].

### 3.5. In Pneumology

There are more than 1.2 million new cases of lung cancer and 1 million deaths occur worldwide every year. At present, the high mortality rate of pulmonary cancer is primarily related to the lack of early diagnosis methods [115]. Accordingly, advanced bronchoscopic diagnostic techniques are playing an increasingly significant role in the detection of lung cancer in recent years [116].

#### 3.5.1. AFI

The role of autofluorescence imaging is majorly investigated in the detection of bronchial premalignant lesions [116–118]. Most of the results confirmed higher sensitivity for the detection of precancerous bronchial lesions when compared to white-light bronchoscopy alone. However, it is known that the specificity of AFI for the detection of premalignant lesions remains low [117].

#### 3.5.2. NBI

As an alternative to AFI in the detection of early lung cancers, NBI has a comparatively higher specificity without significantly compromising the sensitivity [119]. By detecting the surface structure of the lesion and the superficial microvascular morphology of the mucosa, the combination of magnification video bronchoscopy and NBI showed great potential in the detection of precancerous and cancerous lesions of the bronchial mucosa.

#### 3.5.3. FICE

Huang et al. [120] reported that FICE is helpful to observe central type lung cancer. They performed a bronchoscopy examination on 146 patients with the following histologic diagnosis. The coincidence rate of FICE for judging the lesion property was 88.4%. And, the detection rate of FICE combined with WLE for central type lung cancer was 96.6%. Compared with that of single WLE, the detection rate had a statistically significant difference (*P* < 0.01). Also, they revealed that wave combination 8 [*R* = 540 (2), *G* = 505 (4), *B* = 420 (5), wavelength (nm, gain value)] was the most ideal among ten wave combinations in FICE for observing superficial mucosal capillary morphology of pulmonary cancerous tissue.

#### 3.5.4. I-Scan

It was reported that i-scan was able to facilitate the detection of premalignant lesions and early lung cancer [121]. Recently, a prospective multicenter study proposed by Heijden et al. [122] revealed that HD bronchoscopy with i-scan image enhancement was able to detect additional lesions in the central airways. In one-third of all the patients, additional lesions were detected, and their vascular pattern correlated to pathology outcome. However, the interobserver correlation for vascular pattern classification with i-scan was low in their study.

#### 3.5.5. EC

Endocytoscopy owns the potential of in vivo diagnosis of small-cell lung cancer during ongoing bronchoscopy. Shibuya et al. [123] performed probe-based endocytoscopy in twenty-two patients. After the topical application of 0.5% methylene blue, both abnormal regions of interest and normal bronchial mucosa were examined with endocytoscopy at 570-fold magnification. In this study, pEC was useful to discriminate between normal bronchial epithelial cells, dysplastic cells, and malignant cells.

In 2014, Nosaka et al. [124] applied pEC to evaluate the margin and structures of bronchial squamous cell carcinoma in the resected bronchus. This application verified the usefulness of EC for ex vivo histologic diagnosis of the bronchial mucosa. Thus, EC may open a new field of rapid intraoperative diagnosis and shorten the whole operative time. Furthermore, it was reported that pEC had the potential to acquire stable images that are similar to that of conventional hematoxylin or eosin staining and replace intraoperative frozen section examination [125].

However, further studies are needed to validate the diagnostic yield of EC compared with that of standard histopathology.

#### 3.5.6. CLE

The probe-based confocal laser endomicroscopy (*AlveoFlex*, Cellvizio, Mauna Kea Tech) can be applied for *in vivo* microscopic imaging of both upper respiratory tract and distal lung structures during bronchoscopy. CLE makes it possible to detect the semiology of focal and diffuse distal lung diseases. Moreover, CLE can characterize cancerous and precancerous lesions of both upper and distal airways. Thus, CLE is potential to improve endoscopic diagnosis of many lung diseases and to study the lung microcirculation [126].

### 3.6. In Laparoscopic Surgery

Laparoscopic surgery began in the 1980s. Since Dr. Mouret successfully performed the first laparoscopic cholecystectomy in 1987, the application of laparoscopy in clinical surgery has become more and more widespread. Compared with open surgery, laparoscopic surgery has the advantages of “minimally invasive,” such as small incision, unobstructed field of vision, less intraoperative bleeding, less postoperative pain, and faster recovery. Up to now, rigid laparoscopes have been widely used in abdominal surgery (Figure 17), cardiothoracic surgery, urology, gynecology, vascular surgery, and other medical disciplines. Recently, the following advanced optical diagnostic techniques have also been applied to laparoscopy.

#### 3.6.1. UHD-WLE

The continuous improvements of the definition have brought white-light video laparoscopy into a new era. Newly developed CMOS owns an increased number of pixels and increased resolution. In addition, the specialized image processor is used in endoscopy to achieve ultra-high-definition (UHD). Images with 4K UHD (3840 pixels in width and 2160 in height) and 8K UHD (7680 pixels in width and 4320 in height) resolution can be produced to provide four times and eight times more information than conventional Full HD endoscope, respectively [127, 128]. By bringing the UHD endoscope closer to the operative field, minute blood vessels, lymph vessels, and nerves can be distinguished easier, compared with conventional definition images. Because UHD-WLE can shoot a wider range, endoscopists cannot miss any condition in the surrounding areas. Also, immersive experience is created with the help of a bigger monitor compatible with 4K/8K video streaming. Moreover, a wider color gamut was also generated to enable the rich color reproducibility and provide suitable colors for each clinical discipline.

#### 3.6.2. NIR/ICG

Advances in near-infrared (NIR) imaging have expanded the use of fluorescence imaging in endoscopic surgery where detecting structures earlier and differentiating lesions better is essential, due to the use of indocyanine green (ICG), a radioactive, inexpensive fluorescent dye. Alongside an optimal image, NIR/ICG is capable of providing additional information that increases the precision of the surgical operation. Furthermore, NIR/ICG permits the assessment of vascular anastomosis, tissue perfusion, perfusion defects, and identification of lymph nodes. The high penetration depth of NIR light allows visualizing the distribution of ICG up to a depth of 10 mm below the tissue surface.

Since Novadvq's first ICG fluorescent laparoscope was put into clinical practice in 2009, other manufacturers such as the Intuitive, Stryker, and Karl Storz have also launched different types of NIR/ICG laparoscopes into the global market. Recently, OPAL1 technology (Karl Storz) provides a new color option. It allows endoscopists to select the preferred color (green or blue) before or during the procedure. The green color mode offers high-intensity fluorescence with clear differentiation from the surrounding tissue. It additionally achieves a slight optical brightening of the background. In comparison, the blue color mode delivers fluorescence visualization that appears more balanced to the eyes, particularly for the well-perfused liver. Furthermore, the process avoids the potential overexposure of the signals derived from highly fluorescent areas.

NIR/ICG has widespread applications in minimally invasive laparoscopic surgery such as the spermatic vein resection [129], partial adrenalectomy [130], sentinel lymph node biopsy for gynecological tumors [131], and observations of blood perfusion and anastomotic fistula in colorectal cancer [132]. In addition, the system is used to visualize liver metastases or primary tumors of the liver and observe blood perfusion after kidney transplantation in liver surgery [133].

However, the application of ICG fluorescence imaging the liver tumors still has some shortcomings. (i) The detection depth of ICG fluorescence imaging is not enough, and the maximum detection depth is reported to be only 10 mm, so it is impossible to detect deep liver tumors [134]. (ii) The false-positive rate of the examination may reach 40%–50% because the cirrhotic nodules and inflammatory hyperplasia can also emit fluorescence [135].

More recently, the second NIR window fluorescence imaging (NIR-II, 900–1700 nm) has emerged as a highly promising optical imaging technique which has shown many advantages over the clinically available NIR-I imaging (700–900 nm) [136, 137]. These advantages include low level of autofluorescence in the NIR-II region, high signal-to-background ratio, high tissue penetration depth (across centimeters), high in vivo imaging resolution, and larger Stokes shift between emission and excitation light of NIR-II fluorescence [136, 138]. Until now, researchers have founded NIR-II would be a promising imaging technology for intraoperative diagnosis, though none of the commercial NIR-II fluorescence endoscopic system has not been put into clinical use in hospitals. Wu et al. [139] reported that fluorescence cholangiography with ICG in the NIR-II window could provide adequate visualization of the biliary tract structures with increased resolution and penetration depth during cholecystectomy in difficult cases such as cholecystitis patients where obesity and inflammation are quite common, which would result in thickening of the tissue covered on the extrahepatic biliary tract structures. Moreover, Hu et al. [140] proposed an optical-imaging instrument that integrated a visible multispectral imaging system with the detection of NIR-II and NIR-I fluorescence (by using the dye ICG) for aiding the fluorescence-guided surgical resection of primary and metastatic liver tumors. Compared with NIR-I imaging, intraoperative NIR-II imaging provided a higher tumor-detection sensitivity (100% versus 90.6%), a higher tumor-to-normal-liver-tissue signal ratio (5.33 versus 1.45), and an enhanced tumor-detection rate (56.41% versus 46.15%).

Additionally, Suo et al. [136] firstly researched and developed a generalizable-design NIR-II fluorescence endoscopy system, which worked at the subcellular resolution of 20 *µ*m for sharp images in the NIR-II spectra for targeted detection of colorectal cancer. In their study, indocyanine green conjugated bevacizumab (Bev-ICG) that the targeted vascular endothelial growth factor (VEGF) was successfully synthesized and evaluated along with the NIR-II endoscopic system. And, simultaneous NIR-II fluorescence and white-light imaging of VEGF was validated in an orthotopic rat colorectal cancer model.

#### 3.6.3. NBI

By enhancing the visualization of superficial microvascular patterns, NBI is able to characterize lesions with abnormal angiogenesis in the abdominal cavity [141]. Also, NBI was reported to detect more endometriotic lesions. In a study of 167 women who were undergoing pelvic pain or infertility surgery for suspected endometriosis, participants were randomly divided into 3 : 1 ratios between examination by WLE pluses NBI versus WLE alone. Four patients had lesions identified by NBI that were missed by WLE alone, and there was improved sensitivity (100% versus 78.9%) among the 255 histologically confirmed endometriosis lesions sent for pathologic review. The difference in sensitivity for the detection of endometriosis between the two modalities was statistically significant (*P* < 0.001) [142].  Figure 18 illustrates the difference between WLE and NBI.

However, although NBI has been widely integrated into laparoscopes, abdominal surgical applications of NBI need to be continually evaluated. Moreover, the light penetration depth of NBI is less than 1 mm [143], which makes it impossible to identify the lesions deep inside the solid abdominal organs such as the liver and kidney.

#### 3.6.4. EC

In vivo microscopic recognition of malignant lesions in the abdominal cavity can expedite the surgical decision-making process. It was reported that there were two patients undergoing endocytoscopy for intraoperative diagnosis of disseminated malignancy via the laparoscope. Malignant cells in peritoneal nodules were revealed by visualizing the disarray of mitotic cells in the peritoneal mesothelium in vivo, and the diagnostic result was successfully confirmed by the corresponding histopathology. In this way, pEC had the potential to provide on-table diagnosis of presence or absence of peritoneal carcinomatosis [144].

#### 3.6.5. CLE

Probe-based confocal laser endomicroscopy (*CelioFlex UHD 5*, Cellvizio, Mauna Kea Tech) can be used in laparoscopic surgery, and both feasibility and safety of pCLE were confirmed. CLE is currently applied to evaluating the adequacy of laparoscopic liver ablation [145], assessing liver microarchitecture [146], the diagnosis of diversion colitis [147], detections of mucosal changes in ileal pouch after restorative proctocolectomy [148] and the prevention of ovarian cancer [149].

## 4. Future Perspective

Future work related to the advancement of endoscopic imaging may focus on

1. *Increasing the Number of Pixels of Flexible Endoscopes.* At present, the resolution of the rigid endoscopes has reached 4K UHD. It has a high degree of true to life representation while obtaining more detailed information about the targeted area. As a result, 4K UHD rigid endoscopes can be used for delicate neurovascular surgery. Moreover, the field of view of the 4K UHD endoscope is 20 percent larger than before. In the future, flexible endoscopes such as chip-on-tip laparoscopes or gastroscopes may achieve 4K resolution. In this situation, the image quality can be further improved by customizing miniaturized sensors with ITU-R BT.2020 4K standard color gamut and bit depth. However, the greatest challenge now is the design of adequate high-quality lenses.
2. Furthermore, the minimal pixel size is around 0.9–1.0 µm due to the working wavelength; thus, the maximal number of pixels is limited by the space of the distal end of the endoscope, such as ureteroscope or ENT endoscope, where the pixel resolution is limited by small distal diameter.
3. *Probe-Based Endomicroscopy.* For example, probe-based miniaturized optical coherent tomography [150, 151] and two-photon excited fluorescence [152–154] microscopy are promising. With individual administrative approval, the tiny probe can be integrated easily with most therapeutic endoscopes or even work independently to reach specific narrow regions, such as bronchi and bile duct.
4. *Integrating the Wide-Field-View Imaging Techniques with endomicroscopy.* In this way, endoscopists can quickly locate lesions and perform the pathological examination. Thus, the diagnostic accuracy and efficiency can be improved to realize the “one plus one equals more than two” effect. However, it is still unknown which combination of modalities provides the best potential. Thus, more studies are urgently needed.
5. *Computer-Assisted Diagnosis (CAD).* The increasing richness and complexity of medical data have gradually outstripped human analytical capabilities. For example, GI tract cancer has a leading worldwide high incidence and death rate [155]. An estimated 27,510 (17,230 men and 10,280 women) in the United States will be diagnosed with stomach cancer in 2019 [156]. However, the endoscopy is still the golden standard for diagnosing GI tract lesions. It generates massive data owing to the relatively largest internal mucosal surface area and diversely complex diseases. Furthermore, the video data increase even faster when combined with endomicroscopy. Subsequently, it is a heavy burden for clinicians to diagnose during endoscopy. Furthermore, it is impossible to train a doctor with big data that cannot be read within a lifetime. Thus, the emerging of CAD could free the doctor from hard work and help to promote the improvement of endoscopic detection and classification. Hence, CAD can improve the diagnosis accuracy and further reduce the vulnerability of human factors caused by the difference between interobservers.
6. By exploiting the enormous computational power provided by modern computers, CAD algorithms for endoscopic video analysis have already been developed [157–160]. Machine learning offers a technique to recognize informative patterns in large sets of data automatically [161].
7. Recently, studies on CAD algorithms for the detection of colon polyps appeared. For instance, Wang et al. [162] used data from 1,290 patients to develop deep learning algorithms. They validated it on a newly collected 27,113 white-light colonoscopy images from 1,138 patients with at least one detected polyp (per-image sensitivity, 94.38%; per-image specificity, 95.92%). Thus, their result reaches the PIVI threshold presented by ASGE [84]. In addition, the system can process at least 25 frames per second in real-time video analysis with a delay of 76.80 ± 5.60 ms. Hence, the software can aid endoscopists to perform colonoscopy and evaluate the difference in detection performance between polyps and adenomas. However, the algorithm has not yet realized the classification of disease (carcinogenesis, adenoma, hyperplasia, etc.).
8. Based on artificial intelligence, several classification algorithms that combine marketed endoscopic modalities have emerged: such as NBI [163], i-scan [164], and endocytoscopy [165], improving the diagnosis accuracy of GI diseases. In addition, researchers have also developed various CAD algorithms for the detection and diagnosis of esophagus cancer [166], gastric cancer [167], intestinal bleeding [168], and colon tumors [169]. Also, CAD could be utilized in gynecology, such as the diagnosis of uterine fibroids [170] and endometrial cancer [171].
9. Moreover, we believe that CAD is potential to expand the application of optical imaging technologies in the future. For example, with the help of CAD, endocyto may enable rapid scanning and characterizing lesions in a large area of mucosa due to the CAD system has the ability of fast reading. In this way, CAD breaks the limitation caused by the small field of view of EC.
10. Nevertheless, it is essential to note that analytic practices must be used to ensure that the result is robust and valid. This is especially true in health care, for these algorithms have the potential to affect the lives of a large number of patients [172].

## 5. Conclusion

This review intends to provide an accurate and comprehensive synopsis illustrated by a few examples with emphasis on their fundamental principles and actual clinical applications, of where and how clinically available optical diagnostic technologies have already contributed to, or probably will contribute to the way of endoscopic lesion detection and treatment. Thus, this article could serve as a guideline for both biomedical engineers and physicians to increase their understanding in endoscopic optical diagnosis, which is helpful to accelerate a broader range of applications of advanced endoscopic diagnosis technologies in the clinical community and to keep up with state of the art.

As pioneers, clinically available optical imaging techniques have made a considerable contribution to in vivo early detection of subtle abnormalities in many medical specialties, although their compatibilities across specialties are different (Table 3). For example, similar VCE such as NBI and BLI have diverse applications in multiple departments due to various business strategies and administrative regulations. While VCE deals with superficial mucosa lesions, NIR/ICG focuses on specific abnormalities in deeper tissue. Both VCE and fluorescence endoscopy utilize modified spectrums and advanced image processing algorithms to enhance the contrast between lesions and background regions. In addition, UHD-WLE, CF, and DF improve the resolution of visualization under a wide-field of view. Furthermore, EC and CLE provide fundamental insights into mechanisms of human diseases with microscopic images during ongoing endoscopy, thus abolishing the need for random biopsies. Moreover, each technique is seeking self-renewal to strengthen its diagnostic ability. And, with the further development of CAD systems and the maturer integration of CAD algorithms and endoscopic optical imaging platforms, the accuracy and efficiency of disease diagnosis will be greatly improved.

In a word, we believe that the rapid development of endoscopy will lead to a tendency to “all-in-one” for microscopic imaging and functional imaging, which will help endoscopists improve their diagnostic accuracy, especially the detection rate of precancerous lesions. Thus, various research centers are still working on the advancement of endoscopic imaging techniques to prompt the development of healthcare engineering.

## Figures and Tables

**Figure 1:** Overview of the innovative optical imaging technologies applied in existing commercial endoscopes. We classify these techniques into two categories: under a wide field of view or microscopic view. WLE, white-light endoscopy; HD, high-definition; UHD, ultra-high-definition; CF, close focus; DF, dual focus; NBI, narrow band imaging; RDI, red dichromatic imaging; BLI, blue light imaging; FICE, fujinon intelligent chromoendoscopy; SPIES, Storz professional image enhancement system; I-scan OE, i-scan optical enhancement; LCI, linked color imaging; IRI, infra-red imaging; NIR/ICG, near-infrared/indocyanine green; AFI, autofluorescence imaging; PDD, photodynamic diagnosis; EC, endocytoscopy; CLE, confocal laser endomicroscopy; i integrated; p probe-based; e endoscope-based.

**Figure 2:** Brief diagram of the resolution of various types of endoscopes. The imaging resolution of traditional optical fiber endoscopy is determined by the number of optical fibers in its optical fiber bundle. The imaging resolution of flexible electronic endoscopy (such as gastrointestinalscopy) and rigid video endoscopy (such as laparoscopy) has reached 1080p HD and 4K/8K UHD, respectively. SD, standard definition; CCD, charge-coupled devices; CMOS: complementary metal oxide semiconductor.

**Figure 3:** Brief diagram of the correspondence between excitation wavelength and penetration depth. R: red; G: green; B: blue; V: violet; NIR: near-infrared.

**Figure 4:** Timeline for the clinical use of some optical imaging techniques and their corresponding endoscopic systems.

**Figure 5:** The evolution process of available endoscopic tools in gastroenterology. More advanced technologies have been introduced to help endoscopists diagnose gastrointestinal diseases with high efficiency and accuracy. CCD: charge-coupled devices.

**Figure 6:** Schematic diagram of the endoscope working at fixed close focus. Clear visualization of mucosal detail is attained with a larger numerical aperture by shortening the distance between the mucosal surface and the distal end of the endoscope. Thus, more information can be accessed by endoscopists to diagnose accurately.

**Figure 7:** Schematic diagram of the principle of NBI (*EVIS EXERA III*, Olympus, Japan) (e), comparing with white-light imaging (WLI) (a). The spectrum of WLI emitted by a xenon lamp (b) is filtered to become spectrum (c) and spectrum (d), which are the illumination spectrum of WLE and NBI, respectively. The filtered centered wavelengths fall within the peak of hemoglobin absorption bands. Thus, the contrast of mucosal vascular visualization is enhanced to detect lesions accurately. Additionally, the new filter incorporated a mechanism for replacing the red filter with a blue one when systems switch WLE to NBI. Thus, the level of illumination is improved by delivering three flashes of light in every relation rather than just two in the initial generation system.

**Figure 8:** The spectral characteristic of LED narrow-band illumination in NBI mode (460 nm and 540 nm) and RDI mode (540 nm, 600 nm, and 630 nm) activated by Olympus *EVIS X1* system.

**Figure 9:** Schematic diagram of the system of BLI (*ELUXEO*, Fujifilm, Japan). (a) and (d) show the basic principle of WLI mode and BLI mode, respectively. The light source is composed of four LEDs: violet-light LED 1, blue-light LED 2, red-light LED 3, and green-light LED 4. Four paths of light from different directions are compounded into one path by dichroic mirrors, and the thickness of the light path in the diagram represents the actual intensity of each LED light. By adjusting each LED's intensity of radiant emittance, (b) the spectrum of WLE mode and (c) the spectrum of BLI mode can be composited and illuminated on the targeted region. Then, the signals reflected by the mucosa, especially capillary structural signals, are captured by CMOS. Subsequently, they are processed to form an image with higher contrast. LED: light-emitting diode; DM: dichroic mirror.

**Figure 10:** Schematic diagram of SPIES principle. Several specialized modes are capable of enhancing the sharpness of the displayed images and providing specific color renderings. Spectral separation within the RGB camera is amplified by adapted color processing algorithms of the whole spectral light. WLI: white-light imaging.

**Figure 11:** Updates of several virtual chromoendoscopic technologies and their corresponding systems. New-generation techniques are developed to meet the needs of endoscopists and patients better.

**Figure 12:** Brief diagram of the principle of AFI (Olympus, Japan). (a) Green and blue light are generated by a rotating filter, and the spectrum (b) is illuminated to the mucosa. The blue light (400–430 nm) excites endogenous fluorophores in the tissue and emit long-wavelength fluorescence light. (c) The blue light which reflects partially is blocked by the barrier filter, while the excited autofluorescence and reflected green light are finally captured by the CCD. Then, the signal drive from autofluorescence is allocated to the green channel and reflected green light signal is transmitted to another two channels. Hence the images, which represent the normal region in green and the abnormal tissue where there is lack of the autofluorescence signal in magenta or purple in color, are generated to display on the monitor to differentiate lesion and normal area.

**Figure 13:** The spectral characteristic of illumination in WLE mode and IRI (Olympus, Japan).

**Figure 14:** Schematic diagram of confocal microscopy principles. The fluorescence emitted from the focal plane (solid lines) will pass through the pinhole and will be detected. The false fluorescent light emitted from out of focal planes (dashed lines) will be rejected. Illumination source and collection therefore occur in the same focal plane. PMT: photomultiplier tube.

**Figure 15:** Endomicroscopic images of the colon with pCLE (Cellvizio, Mauna KeaTech, France). The field of view of a single image is relatively small, but larger areas can be imaged by merging images from each region. (a) The gray image of the healthy colon mucosa. Arrows indicate dark goblet cells, and clear visualization of regular, round crypt structures are attained. (b) The image reveals adenocarcinoma. Dark and irregularly thickened epithelium (red arrow), disorganized villiform and lack of structure can be viewed.

**Figure 16:** Schematic diagram of currently available two types of confocal laser endomicroscopy. (a) The probe of pCLE can be delivered to be in contact with the tissue through the working channel of endoscopes. Only tissue in the focal plane can be imaged by the mini probe. (b) “Optical sectioning” of eCLE. The eCLE can change the imaging plane depth dynamically during imaging from the surface to the deeper parts of the mucosal layer. (c) The probe.

**Figure 17:** Laparoscopy for liver surgery.

**Figure 18:** Images of tissue near the liver which demonstrate the contrast enhancement provided. (a) WLI image and (b) NBI image.

**Table 1:** Comparison of several contrast-enhancement imaging modalities.

Modality	Illumination (discrete wavelength, nm)		Detection range		
	Band 1	Band 2	Surface	Middle layer	Deeper layer (>10 mm)
NBI	405–425	530–550	✔	✔	✘
RDI	595–600	620–640	✔	✔	✔
AFI	390–470	540–560	✔	✘	✘
IRI	790–820	905–970	✔	✔	✔

Modality	Illumination (continuous wavelength, nm)		Detection range		
	Peak 1	Peak 2	Surface	Middle layer	Deeper layer (>10 mm)

BLI	400	450	✔	✔	✘
i-scan OE	400–450	500–550	✔	✔	✘

**Table 2:** Overview of the advancements and shortcomings of clinically available endoscopic imaging techniques.

Technique	Advancements	Shortcomings
4K/8K UHD	(i) Improving imaging resolution which makes it easier to distinguish minute blood vessels, lymph vessels, nerves, etc. (ii) Shooting with a wider range	Realized in rigid laparoscopy or sinuscopy only
CF	(i) A higher resolving power (ii) Decreasing the minimum visible length to 2 mm	—
Zoom	Enhance surface detail such as pit patterns and vascular detail	The durability of the mechanical zoom system needs further tests
NBI	Improving vascular contrast of capillaries and submucosal vessels based on narrow band light which corresponds to the main and secondary hemoglobin absorption peaks (415 and 540 nm)	The illumination intensity of the 1st generation NBI system is poor
RDI	Enhancing the visibility of blood vessels and bleeding sources in deeper tissue by using narrow band light at two center wavelengths (600 and 630 nm) in the red band	Lacking of further practical clinical experience and data since it has been officially put into clinical use for a very short time
BLI	(i) Highlighting the contrast between blood vessels and surrounding tissues (ii) Enhancing the visualization of relatively distant targets by changing the intensity ratio between blue and violet light (iii) Durable LED light source	Unable to enhance the contrast of submucosal vessels, comparing with NBI
FICE	(i) Providing customized structural and vascular enhancement imaging presets based on spectral image processing algorithm (ii) Better analysis of the pit pattern and the normal-pathological mucosal junction	(i) It is difficult to find the best FICE channels according to different clinical situations (ii) Unstable performance in detecting lesions
SPIES	Five imaging modes are proposed to be candidates according to various clinical situations	Few reports on clinical practice
I-scan OE	Integrating both digital algorithms and optical filters to enhance vascular and mucosal pattern characterization	The technique has just released soon; thus, well-designed clinical trials are warranted and highly anticipated
LCI	(i) Differentiating red color tones more effectively than white-light imaging between the malignant lesion and the surrounding area (ii) Originally red/white regions are represented redder/whiter	Further validation for the diagnosis of malignant lesions is needed
AFI	Detecting neoplastic lesions by exciting endogenous fluorophores such as collagen and flavins in the tissue	(i) Imaging resolution is lower than WLE due to frame averaging, which is utilized to increase the quality of the autofluorescence image (ii) The intensity-based contrast is often not sufficiently specific
IRI, NIR/ICG	Enhancing contrast images of the vessels deep in the mucosa (up to 10 mm)	The false-positive rate of examinations may reach 40%–50% because the cirrhotic nodules and inflammatory hyperplasia can also emit fluorescence
PDD	Improving detection of hardly visible cancer based on the abnormal metabolism of tumor cells in the process of heme synthesis	(i) Phototoxicity of exogenous fluorophores (ii) The validation of the new effective PDD exogenous fluorophores is needed
EC	Visualizing mucosal microstructures in cellular level with high-frame-rate video (30 Hz)	(i) Unable to detect lesions under the mucosal surface (ii) Vital staining is relatively poor (iii) The durability of the ultra-zoom system
CLE	(i) Challenging in-vitro biopsy by identifying structures with cellular and subcellular resolution (ii) Optical sectioning ability	(i) Relatively low frame rate (ii) The interpretation of the acquired image is challenging (iii) Limited lifespan

**Table 3:** Current coverage of clinically available optical imaging techniques in major hospital departments. Most techniques facilitate diagnosis in gastroenterology.

Technique	Gastroenterology (gastrointestinal endoscopy)	Urology (ureteroscopy or cystoscopy)	Gynecology (colposcopy or hysteroscopy)	Otolaryngology (rhinolaryngoscopy)	Pneumology (bronchoscopy)	Laparoscopic surgery
4K UHD				✔		✔
CF	✔	✔	✔	✔	✔	
NBI	✔	✔	✔	✔	✔	✔
RDI	✔					
BLI	✔					
FICE	✔				✔	
SPIES	✔	✔	✔	✔		
I-scan	✔				✔	
LCI	✔					
AFI	✔				✔	
IRI, NIR/ICG	✔					✔
PDD		✔	✔			
EC	✔	✔			✔	✔
CLE	✔	✔			✔	✔

**Table 4:** Comparison of two types of confocal laser endomicroscopy.

Characteristic	Probe-based CLE (pCLE, Mauna Kea Technologies)	Endoscope-based CLE (eCLE, Pentax)	
Scan mode	A single plane	Adjustable planes	
Outer diameter	1.0–2.8 mm	12.8 mm	
Confocal depth	0–70 *μ*m	0–250 *μ*m	
		
Field of view	Ø 240 *μ*m, Ø 325 *μ*m	Ø 500 *μ*m	
Frame rate	9–12 frames/s	0.8–1.6 frames/s	
Spatial resolution	1 *μ*m or 3.5 *μ*m	Lateral	Axial
		0.7 *μ*m	7 *μ*m
